The article "Cardiopulmonary Exercise Testing in the Assessment of Dysfunctional Breathing" was published in 2021. Journal: Front Physiol.

# Cardiopulmonary Exercise Testing in the Assessment of Dysfunctional Breathing

**DOI:** 10.3389/fphys.2020.620955

**Published:** 2021-01-27

**Authors:** Maria F. Ionescu, Sethu Mani-Babu, Luiza H. Degani-Costa, Martin Johnson, Chelliah Paramasivan, Karl Sylvester, Jonathan Fuld

**Affiliations:** ^1^School of Clinical Medicine, University of Cambridge, Cambridge, United Kingdom; ^2^Addenbrooke’s Hospital, Cambridge University Hospitals, Cambridge, United Kingdom; ^3^Hospital Israelita Albert Einstein, São Paulo, Brazil; ^4^Golden Jubilee National Hospital, Clydebank, United Kingdom; ^5^Queen Elizabeth University Hospital, Glasgow, United Kingdom; ^6^Gartnavel General Hospital, Glasgow, United Kingdom; ^7^Royal Papworth Hospital NHS Foundation Trust, Cambridge, United Kingdom

**Keywords:** dysfunctional breathing, breathing pattern disorder, hyperventilation syndrome, CpEt, cardiopulmonary exercise testing

## Abstract

Dysfunctional breathing (DB) is a disabling condition which affects the biomechanical breathing pattern and is challenging to diagnose. It affects individuals in many circumstances, including those without underlying disease who may even be athletic in nature. DB can also aggravate the symptoms of those with established heart or lung conditions. However, it is treatable and individuals have much to gain if it is recognized appropriately. Here we consider the role of cardiopulmonary exercise testing (CPET) in the identification and management of DB. Specifically, we have described the diagnostic criteria and presenting symptoms. We explored the physiology and pathophysiology of DB and physiological consequences in the context of exercise. We have provided examples of its interplay with co-morbidity in other chronic diseases such as asthma, pulmonary hypertension and left heart disease. We have discussed the problems with the current methods of diagnosis and proposed how CPET could improve this. We have provided guidance on how CPET can be used for diagnosis, including consideration of pattern recognition and use of specific data panels. We have considered categorization, e.g., predominant breathing pattern disorder or acute or chronic hyperventilation. We have explored the distinction from gas exchange or ventilation/perfusion abnormalities and described other potential pitfalls, such as false positives and periodic breathing. We have also illustrated an example of a clinical pathway utilizing CPET in the diagnosis and treatment of individuals with suspected DB.

## Background

Dysfunctional breathing (DB) is a collective term used to describe a collection of conditions where the normal biomechanical pattern of breathing is disrupted, resulting in dyspnea and associated non-respiratory symptoms that cannot be fully explained by disease pathophysiology (Barker and Everard, 2015). DB has an overall prevalence of around 9% in the general population but is more prevalent in patients with an underlying respiratory disease, such as asthma or COPD; in asthmatic populations, prevalence has been reported to be as high as 29% (Thomas et al., 2005). There is currently no gold standard diagnosis or classification system and thus the condition is still poorly understood by many clinicians.

The article "Cardiopulmonary Exercise Testing in the Assessment of Dysfunctional Breathing" was published in 2021. Journal: Front Physiol.

When DB was initially described in the literature, a group of symptoms were noted to be associated with inappropriate hyperventilation and over-breathing (Lum, 1975). This was termed hyperventilation syndrome and continues to be a heavily discussed form of DB. However, we now understand this as being just one type of DB as not all patients with DB show hyperventilation responses. More recent literature has looked at the wider picture of DB, with several attempts to classify the different patterns into subtypes (Barker and Everard, 2015; Boulding et al., 2016).

The most important identifying criterion is the presence of breathlessness after organic disease pathology has been ruled out or optimized by pharmacological treatment. This is often described as “disproportionate breathlessness” (Prys-Picard et al., 2006; Barker and Everard, 2015); in other words, the breathlessness is greater than can be ascribed to any potential organic disease. However, as no gold-standard diagnostic method exists, diagnosis is often made using questionnaire-based techniques or following assessment by expert physiotherapists and clinicians.

A major problem with this practice, in our clinical experience, is that symptoms of DB can often be missed or attributed to more severe respiratory disease than there is in reality, resulting in inappropriately high doses of medication that are not beneficial. Identification of DB, on the other hand, would allow patients to benefit from breathing retraining programs delivered by physiotherapists. This will decrease their symptom burden and reduce the need for medication, an overall improvement in their clinical management.

Having said that, we advocate that cardiopulmonary exercise testing (CPET) can be an attractive method to objectively diagnose DB. In that sense, CPET, can identify DB patterns while ruling out other cardiac, respiratory, metabolic and muscular abnormalities (Neder et al., 2018). During CPET, DB often presents with an inappropriately high breathing frequency and erratic patterning of both breathing frequency and tidal volume in response to exercise. Additionally, the patient may report symptoms of DB during the test itself: breathlessness at a low workload, chest tightness, dizziness or tingling sensations in their lips and/or fingers.

The article "Cardiopulmonary Exercise Testing in the Assessment of Dysfunctional Breathing" was published in 2021. Journal: Front Physiol.

This review focusses on the pathophysiology and proposed tests to diagnose DB, followed by a brief discussion on how such tests might aid in planning personalized patient care. It is important to note that, despite the growing interest in DB in recent years, published research evidence that supports our understanding of the condition is limited. Thus, some of the information provided and discussed here comes from expert opinion and clinical experiences, as well as research published only in abstract form.

## Pathophysiology of Dysfunctional Breathing

Dysfunctional breathing encompasses any change in the normal biomechanical pattern of breathing; within this, there have been attempts to classify DB into subtypes. Barker and Everard suggested a classification system which splits DB into thoracic (alterations in the respiratory muscle activity) or extra-thoracic (with upper airway involvement too). The thoracic and extra-thoracic types were then each further split into structural and functional subtypes (Barker and Everard, 2015; Depiazzi and Everard, 2016). Within thoracic DB, Boulding and colleagues proposed a classification system largely based on the pathophysiological pattern of disruption to the respiratory muscle activation, identifying five key types of DB: hyperventilation syndrome, periodic deep sighing, thoracic dominant breathing, forced abdominal expiration and thoraco-abdominal asynchrony (Boulding et al., 2016).

Thoracic and extra-thoracic DB are diagnosed and managed differently in clinical practice. For the purposes of this manuscript, we have focused on the thoracic types of DB, as CPET is useful for their identification. However, it is important to be aware of the subclassifications which exist within DB.

Regarding the pathophysiology of thoracic DB, it is often physiological or psychological stress which provokes symptoms (Depiazzi and Everard, 2016). These stressful events can include excessive aerobic training, bereavement or a health-related illness (Courtney, 2009). Respiratory diseases (such as asthma or COPD) as well as musculoskeletal dysfunction, pain or an altered chest wall shape can also cause DB, by triggering the diaphragm into an abnormal pattern of breathing (Barker and Everard, 2015; Berton et al., 2020).

Fluoroscopic studies have demonstrated that when an individual is exposed to emotional stress the diaphragm becomes flattened, hypertonic and relatively immobile, causing intercostal and accessory muscles to contribute more to ventilation (Courtney, 2009). This is associated with mild hyperinflation, an irregular rate and volume of respiration and frequent sighing. DB can therefore be seen as an unconsciously learned habitual change in the normal pattern of breathing which may become apparent at rest or only when stressed (Barker and Everard, 2015). In some patients, there is a sufficient increase in minute ventilation to cause hypocapnia. This occurs for varying lengths of time, depending on the cause. However, only a small proportion of patients with thoracic DB exhibit hyperventilation as defined by the presence of hypocapnia.

The article "Cardiopulmonary Exercise Testing in the Assessment of Dysfunctional Breathing" was published in 2021. Journal: Front Physiol.

A certain level of hyperventilation may be associated with increased sympathetic activity when stressed, which has the potential beneficial effect of increasing neuronal activity. However excessive sympathetic activity with further hyperventilation and hypocapnia results in the depression of neuronal activity. Overall it has been shown that exercise has a greater effect on respiratory volumes in comparison to anxiety, which is associated more with irregular breathing (Barker and Everard, 2015).

Extra-thoracic subtypes of DB have a different pathophysiology, characterized by upper airway changes (Barker and Everard, 2015; Depiazzi and Everard, 2016). The most common of these extra-thoracic changes are inducible laryngeal obstruction (ILO) and laryngomalacia. ILO is the intermittent, abnormal, paradoxical adduction of the vocal folds with respiration, causing variable upper airway obstruction (Krey and Best, 2014; Matrka, 2014; Halvorsen et al., 2017). In laryngomalacia there is intermittent airway obstruction due to collapse of the supraglottic tissues during inspiration when an individual is exercising vigorously and generating large negative intrathoracic pressures (Shembel et al., 2017). It is also possible that the changes to the diaphragm seen on fluoroscopic studies also occur in the glottis leading to paradoxical vocal fold dysfunction.

## Diagnosis Methods

There are a wide range of diagnostic methods in use in clinics today. However, there is no gold-standard, validated method being consistently applied. Centers utilize different strategies which unfortunately do not show complete overlap in the diagnoses picked up by the different methods (Todd et al., 2018).

Questionnaire-based approaches, such as the Nijmegen questionnaire (NQ) and the self-evaluation of breathing questionnaire (SEBQ), are common methods used to identify DB. The NQ is the most widespread method, despite only being designed to identify hyperventilation syndrome. It utilizes a series of questions to identify how frequently a patient experiences certain symptoms, assigns each response a score of 0–4 and a total NQ score is calculated. If this NQ score is above the threshold of 23, a DB diagnosis can be considered likely.

The article "Cardiopulmonary Exercise Testing in the Assessment of Dysfunctional Breathing" was published in 2021. Journal: Front Physiol.

The NQ was found to have a sensitivity of 91% and specificity of 95% in detecting hyperventilation (van Dixhoorn and Duivenvoorden, 1985); the submaximal sensitivity was proposed to be due the questionnaire using an incomplete list of symptoms and thus missing some patients with unusual sets of symptoms. Alternatively, patients may not necessarily notice or report their own symptoms as abnormal, which would also result in the questionnaire failing to detect the hyperventilation. In the context of subjects with other conditions, such as poorly managed asthma, COPD, panic disorder and anxiety, the specificity of the NQ is lower due to an inability to distinguishing DB from underlying co-morbidities (Stanton et al., 2008; van Dixhoorn and Folgering, 2015). Thus, it has been proposed that the NQ represents a subjective score of “functional respiratory complaints” that may point to but not be unique to DB or hyperventilation (van Dixhoorn and Folgering, 2015).

Other diagnostic methods utilize direct observation and examination by expert physiotherapists. Physiotherapists can use a tool such as the Breathing pattern assessment tool (BPAT) (Todd et al., 2018) or the manual assessment of respiratory motion (MARM) method (Courtney et al., 2008). The benefit of these methods is that the assessment of the breathing pattern is made by an observer, rather than relying on patient-reported symptoms. Moreover, an expert physiotherapist specializing in this field can rapidly make an assessment of the breathing mechanics; they are able to pick up on visual and physical clues and utilize pattern recognition to help to make the diagnosis. A potential difficulty is that it requires expert chest physiotherapists familiar with DB and the observational and analytic skills require frequent exposure to DB to build up. Thus, it may not be possible to put this into practice in all centers.

A less frequently used method which can be used in the diagnosis of DB is plethysmography, either optoelectronic or inductive. These methods rely on measuring the changes in volume of the chest wall, ribcage and abdomen in order to analyze the underlying breathing mechanics. This has the potential to be a sensitive technique to study thoracic-dominant DB or thoracic-abdominal asynchrony. Despite its current limited clinical use, literature has supported that plethysmography may be a useful tool to characterize breathing patterns (Levai et al., 2016).

Finally, ramp-incremental CPET can be very helpful for the investigation of dyspnea of unknown etiology. It allows identification of any pathophysiological cause of breathlessness on exertion which could not be demonstrated by tests performed at rest. In that sense, aerobic, ventilatory, cardiac, gas exchange and muscle response to exercise can be determined and compared to normal predicted responses (Wasserman, 1997). Thus, it is an attractive method by which to identify DB clinically (Toma et al., 2010; Griffiths and Anindo, 2014; Costa et al., 2016; Jayadev et al., 2017; Roberts et al., 2017; Brat et al., 2019).

The article "Cardiopulmonary Exercise Testing in the Assessment of Dysfunctional Breathing" was published in 2021. Journal: Front Physiol.

The CPET begins with a resting phase analysis of the patient’s spirometry, ECG, blood pressure and oxygen saturation. For some patients, DB may be apparent at rest. The patient is asked to quantify their feeling of breathlessness and muscle fatigue at the start of the test, measures which will be revisited at the end of the test. Additionally, an evaluation is made of the subject’s functional status and baseline level of fitness, enabling the physiologist to estimate a predicted workload ramp rate to use during the test. Subsequently, the exercise test proceeds to the exercise phase of the test, typically carried out on a stationary bike. This begins with unloaded cycling, followed by incrementally increased load until the patient is stopped by symptoms or the physiologist stops the test due to safety concerns. Ideally this maximal exertion should be reached after about 8–12 min of loaded exercise. The patient’s physiological response to exercise is monitored throughout the exercise and subsequent recovery, until the patient returns back to their baseline. At peak exercise, the patient is asked to quantify their feeling of breathlessness and muscle fatigue. In patients with DB, the factor leading to cessation of exercise will often be sensations of breathlessness or air hunger due to the inefficient breathing pattern. A standard CPET protocol has been described in detail in the European Respiratory Society’s statement on standardization of CPET testing in chronic lung diseases (Radtke et al., 2019).

The literature in the CPET field is heavily weighted toward stationary cycle ergometers as the exercise modality of choice. In practice, it would be possible to apply an incrementally increasing workload using other modalities, such as treadmills or indoor rowing machines. For instance, treadmills are the exercise method utilized in the Bruce protocol, which is typically used for exercise stress tests in the context of cardiology (Bruce et al., 2004). Alternative exercise modalities could be particularly useful for athletic individuals, providing a method to analyze their physiological response to exercise in a scenario that is closer to their typical training regime. This suggestion has been made in the literature for cardiology stress tests (Sarma and Levine, 2016). Use of the Bruce protocol or alternative exercise modality has not been described in the literature for the purposes of DB, but it is possible that a similar approach could be utilized.

The article "Cardiopulmonary Exercise Testing in the Assessment of Dysfunctional Breathing" was published in 2021. Journal: Front Physiol.

A major benefit of CPET is that, unlike the questionnaires and observation-based approaches, it gives objective measurements and plots data which can be directly analyzed. The nine-panel plot provides an excellent visual method to analyze these data. Erratic or abnormal responses in the respiratory panels can point to a diagnosis of DB. This will be discussed in further depth in the next section. Moreover, CPET can help to rule out other causes of exercise limitation. The cardiac panels, ECG and metabolic analysis can exclude other pathologies or drivers to DB. As discussed, this is a vital step in making a diagnosis of DB. CPET can provide reassurance that there is no underlying disease pathology, helping to confirm whether DB is the main cause of a patient’s symptoms (Toma et al., 2010; Costa et al., 2016).

The use of CPET to aid in the diagnosis of patients with unexplained dyspnea has been supported in recent literature. A proportion of these patients were found to have DB upon analysis of CPET data (Thing et al., 2011). This, however, is likely to be an underestimate, as we would argue that DB is still underdiagnosed by most clinicians. This underdiagnosis probably stems from the lack of a consistent definition and classification system. Hyperventilation syndrome remains the most widely discussed type of DB, but it should not be taken to be synonymous with DB. Unfortunately, many clinicians are not familiar enough with the different types of DB to identify the rarer types that do not present with hyperventilation.

## CPET Data Interpretation

Using maximal ramp-incremental CPET to rule out other causes of breathlessness is important when investigating DB, as DB is sometimes a diagnosis of exclusion. It may also be very reassuring to patients to know that there is no obvious underlying disease process.

The first step in interpreting the results of a CPET is pattern recognition using techniques such as the 9-panel plot. The nine-panel plot gives a useful overview of the aerobic, ventilatory, cardiac, gas exchange, and muscle response to exercise, which can be used to suggest the presence, severity and relevance of any pathophysiology. If there is no disease pathophysiology detected, or the degree of symptoms exceed what would be expected from the pathophysiology, this may suggest an element of DB.

There are different approaches when analysing CPET results. We recommend standardizing the reading according to the following steps: (Barker and Everard, 2015) check that the test fulfils criteria for maximum effort; (Thomas et al., 2005) analyze the physiologic responses to exercise, moving sequentially from metabolic responses, to cardiovascular responses and finally to ventilatory and gas exchange responses; (Lum, 1975) assess causes for stopping exercise (dyspnea and/or leg discomfort) and other potential accompanying symptoms such as light headedness, chest pain or perioral numbness. Here we describe what physicians should expect to encounter at each of these steps when exercise intolerance is due to DB. It should be stressed that some of the information provided below is derived from expert opinion and clinical experience, but appropriate research papers are referenced when the evidence is available.

1. Checking criteria for maximum effort
Patients with DB may not fulfill the usual criteria for maximum effort. It is not uncommon for them to stop exercising at heart rates which fall below 85% of the predicted maximal, usually at low work rates (Figure 1A) and showing additional evidences of submaximal test. The respiratory exchange ratio (RER) at peak exercise, on the other hand, can be lower or higher than 1 depending on the breathing pattern the patient assumes during exercise. Patients who develop significant hyperventilation may start and finish exercise with RER values persistently above 1 (Neder et al., 2018). Conversely, development of an erratic ventilatory pattern may result in tremendous unpredictable variations of its value over time, so that RER at peak exercise may fall randomly below 1 (Figures 1B,C).

The article "Cardiopulmonary Exercise Testing in the Assessment of Dysfunctional Breathing" was published in 2021. Journal: Front Physiol.

**FIGURE 1:** Example 9-panel plot showing patterns consistent with DB. The panels give an overview of metabolic **(A,C)**, cardiovascular **(D,G)**, ventilatory **(B,E,F,H)** and gas exchange **(I)** responses during the CPET. VO2, volume of O_2_ used per minute; VCO2, volume of CO2 produced per minute; VE, minute ventilation; BTPS, body temperature and standard pressure; HR, heart rate, VE/VCO2, ventilatory equivalent for CO_2_; VE/VO2, ventilatory equivalent for O_2_. PETCO2, end-tidal CO_2_; PETO2, end-tidal O_2_.

2. Analysis of physiologic responses to exercise
a. Metabolic responses
Patients with DB might present with normal or reduced VO_2_ at peak exercise (MartinezI, 1994; Chenivesse et al., 2014; Brat et al., 2019). In the latter case, it is not uncommon for the test not to fulfill criteria of maximum effort. The anaerobic threshold (AT) might be difficult or even impossible to determine in cases were erratic ventilation develops, as the ventilatory equivalents become too variable and unpredictable over time (Figure 1F). Also, the AT may not be reached if patients stop exercising prematurely. However, when AT is present and identifiable, the VO_2_ is expected to be within the normal range (MartinezI, 1994). The VO_2_/W slope is usually (although not always - Figure 1A) possible to estimate and is expected to be within the normal range as well.
b. Cardiovascular responses
Patients with exercise intolerance due to DB are expected to have normal cardiovascular responses to exercise. In that sense, HR, arterial pressure and oxygen pulse should increase appropriately with progressively higher exercise intensities. For most patients, peak HR is higher than 85% of the predicted maximal (MartinezI, 1994; Brat et al., 2019), but lower peak HR can be seen in the context of submaximal effort. Having said that, it is important to analyze submaximal variables such as HR/VO_2_ slope, as they are expected to remain in the normal range even if exercise is stopped prematurely (Figure 1D).
Oxygen pulse (VO_2_/HR) is yet another important variable to assess, as it is considered a surrogate for stroke volume and is generally reduced in cardiovascular and pulmonary vascular disease (Degani-Costa et al., 2019). In patients with DB, O_2_ pulse at peak exercise is expected to be normal (MartinezI, 1994), but development of erratic breathing might make it difficult to analyze its submaximal trajectory or even determine its peak value accurately. The more erratic the ventilation, the more scattered averaged VO_2_/HR values become, even if the data is adequately smoothed (Figure 1G).
c. Ventilatory and gas exchange responses
The ventilatory and gas exchange variables are the ones that can be most informative to distinguish DB from other causes of exercise intolerance. In healthy individuals, increments in ventilation (*V*_*E*_) during the early phases of exercise are primarily due to an increase in *V*_*t*_, with minimal increases in *B*_*f*_ (Figures 2A,B). As the subject faces progressively higher workloads, *V*_*t*_ plateaus and further increments in ventilation become strongly dependent on the rise of *B*_*f*_. This physiological response minimizes dead space (*V*_*D*_/*V*_*T*_) and allows *V*_*E*_ to increase linearly (and predictably) with carbon dioxide production (*V*_*CO*__2_) throughout the greater part of loaded exercise, until the *V*_*E*_/*V*_*CO*__2_ slope demonstrates an inflection as the respiratory compensation point is reached (Wasserman, 1997; Neder et al., 2003).

The article "Cardiopulmonary Exercise Testing in the Assessment of Dysfunctional Breathing" was published in 2021. Journal: Front Physiol.

**FIGURE 2:** Illustrative plots of breathing frequency (labeled as BF on left *y*-axis) and tidal volume (labeled as VTex on right *y*-axis) against minute ventilation (labeled as V’E on *x*-axis), showing breathing pattern responses to ramp-incremental CPET in five possible scenarios. Such plots allow for greater insight into the breathing pattern over the course of the CPET, looking at both *V*_*t*_ and B_*f*_ changes with ventilation. The five scenarios illustrated are: **(A)** normal individual **(B)** athletic individual **(C)** early DB that resolves on exercise **(D)** DB manifesting upon commencement of exercise **(E)** DB throughout. Particular attention should be paid to the predictable pattern of breathing frequency and tidal volume increases in plots **(A,B)**, allowing for an efficient mechanism for minute ventilation to increase; this can be contrasted to the erratic patterns that can be observed in plots **(C–E)**, which are indicative of DB. BF, breathing frequency; V’E, minute ventilation; VTex, tidal volume.

On the other hand, patients with DB usually present with high *B*_*f*_ at rest which increases inappropriately quickly in early exercise, while *V*_*t*_ may remain essentially unchanged. This can increase dead space ventilation and alter the kinetics of many CPET variables (Neder et al., 2016), typically increasing *V_E_*/*V*_*CO*2_ slope (Figure 1E). Also, this rapid shallow breathing pattern, characteristic of hyperventilation syndrome, may result in increased end-inspiratory and end-expiratory lung volumes, therefore reducing inspiratory capacity and possibly contributing to the unpleasant dyspnea sensation irrespective of the occurrence of true hypocapnia (Boulding et al., 2016).
In many cases, however, frequent sighing also occurs in the middle of this rapid shallow breathing, generating a chaotic and irregular breathing pattern (Boulding et al., 2016), with highly variable *V*_*t*_ and *B*_*f*_ for a given *V*_*E*_. When this occurs, the impact of the breathing pattern on operating lung volumes is poorly understood, as it is virtually impossible to perform inspiratory capacity maneuvers correctly without ensuring regular and stable *V*_*t*_.
Such DB patterns (hyperventilation, erratic ventilation and/or periodic sighing) may disappear later in exercise as the subject becomes more focused on the task (Figure 2C) or, on occasions, only begin only after the patient starts pedaling (Figure 2D). In some cases, though, they persist throughout the whole test (Figures 1H, 2E). Since CPET collects both resting and exercise data, all of these patterns of DB can be identified. DB that only becomes obvious on exertion can be missed by other clinical assessment methods.
While identification of erratic ventilation may seem rather straightforward at first, in practice many cases can pose a significant challenge. Given the irregular and unpredictable nature of this ventilatory pattern (which clearly distinguishes it from periodic breathing), to date no objective, measurable and standardized criteria have been developed to define it. As such, the diagnosis of erratic ventilation requires the utilization of pattern recognition skills of the clinician interpreting the CPET data. In our experience, looking at a few specific plots can be helpful: (1) *V*_*E*_/*V*_*O*__2_ and *V*_*E*_/*V*_*CO*__2_ against time; (2) P_*ET*_CO_2_ and P_*ET*_O_2_ against time; (3) *B*_*f*_ and *V*_*t*_ against time; (4) *B*_*f*_ and *V*_*t*_ against *V*_*E*_. On these plots, the respiratory equivalents, P_*ET*_CO_2_ and P_*ET*_O_2_ show irregular and erratic kinetics (Figures 1F,I) and *B*_*f*_ and *V*_*t*_ data points appear scattered rather than linear (Figures 1H, 2E). Of course, this analysis depends on adequate smoothing of the data, and either moving average of eight breaths or running average of five of seven breaths can be used. Still, identifying erratic ventilation can be rather subjective in some cases.
Previous authors have attempted to propose strategies for pattern recognition and cut-offs for gas exchange variables which could reliably identify DB on CPET. More specifically, Boulding and colleagues proposed classifying DB patterns taking into account not only incremental CPET data, but also the behavior of *B*_*f*_, *V*_*t*_, and respiratory muscle mechanics before and after exercise (Boulding et al., 2016). By that approach, in addition to hyperventilation syndrome and erratic ventilation, other abnormal breathing patterns might be identified: thoracic dominant breathing, forced expiratory pattern and thoraco-abdominal asynchrony. Thoracic dominant breathing pattern was characterized by a lack of costal expansion and a high reliance on upper thoracic muscles during inspiration. As with hyperventilation, thoracic dominant pattern was associated with high operating lung volumes and reduced inspiratory capacity. The forced-expiratory pattern, on the other hand, results in the patient breathing on very low lung volumes, therefore reducing functional residual capacity.
However, the inherent caveats of CPET data interpretation make it usually impossible to rely solely on breathing patterns to establish a diagnosis of DB. For instance, thoracic-dominant and forced expiratory breathing patterns may develop in patients with COPD in response to pulmonary hyperinflation, in which case they should not be regarded as dysfunctional, but rather as a physiological adaptation. Similarly, thoracic-dominant patterns may be seen in morbidly obese patients in response to their low abdominal compliance. Finally, significant hyperventilation may occur in patients with increased dead space ventilation, such as those with heart failure or pulmonary hypertension.
Therefore, in patients undergoing CPET for unexplained dyspnea who present with abnormal breathing patterns, additional physiological information (summarized in Table 1) must be analyzed before establishing any diagnosis, as certain cardiac or respiratory pathologies can present similarly to DB on CPET. First of all, patients with purely DB generally stop exercising with a high breathing reserve, although ventilation is clearly dissociated from the metabolic demand (Neder et al., 2018). Second, patients are not expected to desaturate during exercise, unlike patients with lung parenchyma and pulmonary vascular disease. Importantly, arterial or capillary blood gases at rest and peak exercise can also help discriminate DB from cardiopulmonary conditions. In that sense, patients with DB usually present with resting hypocapnia and normal PaO_2_, P(A-a)O_2_ gradient, *V*_*D*_/*V*_*T*_ and P(a-ET)CO_2_ gradient at end-exercise, which can help differentiate from other conditions in which chronic hyperventilation occurs, such as heart failure or PAH.

The article "Cardiopulmonary Exercise Testing in the Assessment of Dysfunctional Breathing" was published in 2021. Journal: Front Physiol.

**TABLE 1:** Summary of typical blood gas and CPET findings in DB compared to other diseases.

	**Dysfunctional breathing (DB)**	**Left heart disease (without PAH)**	**Pulmonary arterial hypertension (PAH)**	**Interstitial lung disease (ILD)**	**COPD**
PaCO_2_ at rest	Normal or low	Normal to low	Low	Normal	Normal or high
PaO_2_ at end-exercise	High or normal	Normal	Low	Low	Normal
P(A-a)O_2_ gradient	Normal	Normal	High	High	Normal
P_*ET*_CO_2_ at AT or end exercise	Typically low	Normal to low	Very low	Normal to low	Normal to high
*V*_*E*_/*V*_*CO2*_ slope	Typically high	Normal to high	Very high	High	GOLD I-II: High GOLD III-IV: normal to low
P(a-ET)CO_2_ gradient	Normal but can be high	Normal	High	High	High
*V*_*D*_/*V*_*t*_	Normal but can be high	Normal	High	High	High

*The conditions below have been highlighted as clinical scenarios that may present similarly on CPET, but can be distinguished from DB by using the parameters detailed in the table. PaCO_2_, arterial partial pressure of CO; PaO_2_, arterial partial pressure of O_2_; P(A-a)O_2_ gradient, alveolar-arterial gradient of O_2_; P_*ET*_CO_2_, end-tidal partial pressure of CO_2_; AT, anaerobic threshold; *V*_*E*_, minute ventilation; *V*_*CO2*_, volume of CO_2_ exhaled per minute; P(a-ET)CO2, arterial – end-tidal CO_2_ gradient; *V*_*D*_, dead volume; *V*_*t*_, tidal volume.*

Conversely, while resting P_*ET*_CO_2_ below 30 mmHg, unchanging P_*ET*_CO_2_ and VeqCO_2_ or an inverse trend of P_*ET*_CO_2_ and VeqCO_2_ kinetics during loaded exercise (i.e., early decrease in P_*ET*_CO_2_ and increase in VeqCO_2_ rather than the opposite) have been suggested as highly specific of primary hyperventilation syndrome, a similar pattern can also be seen in patients with pulmonary arterial hypertension (Brat et al., 2019).
It should be noted that the presence of erratic ventilation does not automatically exclude alternative clinical diagnoses. DB frequently coexists with asthma and is recognized as a cause of severe and difficult-to-treat asthma (Boulding et al., 2016). Also, patients with a history of stridor or those who develop stridor during the test should be investigated for vocal cord dysfunction. On the other hand, there is no specific recommendation to treat DB when erratic ventilation is an incidental finding and the patient is asymptomatic. Of course, since CPET is usually performed as a diagnostic test to identify a cause of dyspnea in patients who are symptomatic, identification of DB in these patients is likely to be of clinical significance.
Finally, it is important to consider particular differentials of erratic ventilation, such as pulmonary arterial hypertension or periodic breathing associated with heart failure. These conditions may also present with an “erratic-looking” *B*_*f*_ and *V*_*t*_ plots, but as described above it is possible to use further CPET plots and variables to distinguish between these two entities (Figure 3). Similarly, periodic breathing can be readily distinguished from DB by carefully analysing nine-panel plots, particularly the one portraying *V*_*E*_ over time. Periodic breathing is a recognized marker of disease severity in patients with heart failure due to left ventricular systolic dysfunction and may develop at rest or during exercise. As happens in DB, periodic breathing may last throughout the whole phase of incremental workload or disappear toward the end of exercise. However, the characteristic periodicity of waxing and waning of *V*_*t*_ (and consequently of *V*_*E*_) seen in periodic breathing (Agostoni et al., 2017) is in clear contrast to the unpredictable and irregular breathing pattern of DB (Figures 3A,B,D,E). Given its predictable behaviour, standardized criteria have been adopted to define periodic breathing, the most widely accepted one requiring the amplitude of a single *V*_*E*_ oscillation to be greater or equal to 15% of the resting average *V*_*E*_ and the phenomenon to last at least 60% of the exercise phase (Agostoni et al., 2017).

The article "Cardiopulmonary Exercise Testing in the Assessment of Dysfunctional Breathing" was published in 2021. Journal: Front Physiol.

**FIGURE 3:** Representative CPET plots that can be used to help distinguish between DB, pulmonary arterial hypertension and heart failure with periodic breathing. These conditions may be differentials in patients undergoing CPET for unexplained dyspnea suspected to be DB All three may present with seemingly erratic patterns of *V*_*t*_ and B_*f*_ responses to exercise. Therefore these plots can be used to narrow down the diagnosis when interpreting a CPET. Note that in columns 1 and 2 the colors on the *x*-axis indicate the phase of exercise; gray is rest, green is unloaded cycling red is linearly increasing workload and yellow is recovery. In the third column, unloaded cycling began at 2 min and loaded cycling at 5 min. **(A)** Plot of minute ventilation and oxygen saturation against time. **(B)** Plot of minute ventilation against volume of CO_2_ exhaled per minute. **(C)** Plot of ventilatory equivalents for CO_2_ and O_2_ against time. **(D)** Plot of respiratory exchange ratio against time. **(E)** Plot of end-tidal CO_2_ and O_2_ against time. Particular points to take from this figure are the similarity in appearance of DB and pulmonary arterial hypertension plots. Major differences include the desaturation in pulmonary arterial hypertension and the fall in respiratory exchange ratio in later exercise in DB. Additionally, note the clear periodicity across the plots in the case of heart failure with periodic breathing; this is not the case for DB. *V*_*E*_, minute ventilation; SpO_2_, oxygen saturation; *V*_*E*_/*V*_*CO2*_ or VeqCO_2_, ventilatory equivalent for CO_2_; *V*_*E*_/*V*_*O2*_ or VeqO_2_, ventilatory equivalent for O_2_; P_*ET*_CO_2_, end-tidal CO_2_; P_*ET*_O_2_, end-tidal O_2_; RER, respiratory exchange ratio; RCP, respiratory compensation point; Vth1, first ventilatory threshold; VO_2_max, point of maximal O_2_ consumption; AT, anaerobic threshold.

d. Reasons for stopping exercise and accompanying symptoms
Enquiring after the reasons for stopping the test and accompanying symptoms can also aid in differentiating between DB and other clinical conditions. For example, the development of perioral numbness, tingling and peripheral paraesthesia is highly suggestive of DB and a dissociation between dyspnea intensity and the workload level can also be seen (Neder et al., 2016).

## CPET as a Guide to Treatment

Dysfunctional breathing is usually very responsive to breathing retraining by specialized physiotherapists (Thomas et al., 2003). In our clinic, we provide follow-ups after the initial assessment visit, where patient progress can be tracked. If the patient can consciously control their breathing pattern at follow-up, the next step is to try to perform the same breathing pattern in a more challenging scenario, for instance when walking along a corridor, going up and down stairs, or having a conversation. This will help them train the new way of breathing to become subconscious. There is no published data describing the role of CPET in guiding individual therapy.

The article "Cardiopulmonary Exercise Testing in the Assessment of Dysfunctional Breathing" was published in 2021. Journal: Front Physiol.

Educating patients about DB is a key component and first step in the breathing retraining program. In this context, CPET can help patients and clinicians by reassuring them that dyspnea is not the result of an underlying organic pathology, Furthermore, the modified Vt and Bf plot guides the clinician to understand the variance in the breathing pattern and adds a degree of objectiveness to their assessment of the breathing pattern. Showing the patient this plot can also provide visual feedback to the patient about the changes in their breathing pattern, which then allows the clinician to promote awareness of the effective breathing pattern and improve patient engagement with breathing retraining.

Over the course of the therapy, progress from the initial assessment to subsequent visits is often tracked using NQ, SEBQ, or BPAT scores. As discussed before, these are quite subjective methods to assess symptoms and breathing pattern. Moreover, when used as a method to monitor progress, they can also risk being biased. If the questionnaire is being filled out by a patient, they know they are undergoing therapy, and may try to, either consciously or subconsciously, answer the questions as they think the practitioner wants them to, decreasing the scores given to describe the frequency of their symptoms to show the treatment working. Importantly, the physiotherapist or other assessing practitioner may themselves show a certain degree of bias in the follow-up assessments, since they know that the patient has had therapy and so will be looking to see that this therapy has worked.

In reality, it has been observed that patient symptoms and quality of life improve even if the NQ/SEBQ/BPAT scores do not show a significant change from the baseline. Thus, perhaps we have been going about trying to quantify the degree of breathing pattern change incorrectly. Indeed, Thomas and colleagues identified that the change in the AQLQ score (a questionnaire aimed to quantify asthma-related quality of life) showed a more significant response to breathing retraining in asthmatics with DB compared to the NQ score (Thomas et al., 2003).

Cardiopulmonary exercise testing may be useful as an objective assessment tool, to guide the process of breathing retraining and monitor the progress over the course of therapy. Comparing a patient’s CPET data before and after therapy could provide objective support that the breathing retraining therapy is having a beneficial effect. Problems may arise in terms of CPET availability, limiting the extent to which this modality could be used to monitor patients’ progress.

The article "Cardiopulmonary Exercise Testing in the Assessment of Dysfunctional Breathing" was published in 2021. Journal: Front Physiol.

## Key Messages

Dysfunctional breathing is a condition which is variably classified and lacks a standardized investigation and management approach. This paper highlights the many disparate methods used to diagnose DB, consequent on the lack of consensus on how best to diagnose the condition (van Dixhoorn and Folgering, 2015; Todd et al., 2018). In order to alleviate this confusion, it is important that there is a single clear definition of DB with one classification system. There also needs to be a single objective test which can analyze and define erratic ventilation in order to diagnose DB. Creating these standards will make it easier to identify and manage the condition.

Cardiopulmonary exercise testing represents a particular opportunity to objectively assess different aspects of individuals’ physiology, particularly the presence of underlying organic disease and/or evidence of erratic ventilation (Costa et al., 2016). Thus, CPET is an ideal candidate to be the standard objective diagnostic method for DB.

A key component of identifying DB using CPET is recognizing the abnormal erratic breathing pattern response to exercise. This is not a parameter that can be easily quantified, and as such, there is no absolute diagnostic threshold. However, clinicians’ use of pattern recognition when analysing the Bf and *V*_*t*_ plot is of high importance. This can be supplemented by using the further CPET variables highlighted. A low P_*ET*_CO_2_ at rest or during work (Brat et al., 2019) and a high VeqCO_2_ during work (Kinnula and Sovijarvi, 1993; Brat et al., 2019) in the absence of desaturation are particularly suggestive of DB. Suggested cut-off values for these parameters have been proposed in the literature: a P_*ET*_CO_2_ below 30 mmHg at rest or during work (Brat et al., 2019) and a VeqCO_2_ above 35 at a workload of 40–50 W (Kinnula and Sovijarvi, 1993) may help to make the diagnosis of DB. However, it is not as straightforward as having diagnostic thresholds beyond which a diagnosis can be definitively made. These CPET data should be interpreted in the context of other investigations, such as blood gas readings, to provide the entire clinical picture for the diagnosis of DB.

Nevertheless, CPET is not a perfect tool. Since it is just a snapshot into the subject’s physiology for 20–40 min, a major problem is that patients may not always manifest DB during the test. Patients with a constant DB pattern or whose DB is strongly linked to exertion are easily picked up by CPET, but patients who only occasionally exhibit DB may be missed, resulting in false negatives. Similarly, upper airway abnormalities, such as laryngeal disorders, commonly present with exertional breathlessness and require specific investigations such as laryngoscopy during exercise for their identification (Hull et al., 2016).

The article "Cardiopulmonary Exercise Testing in the Assessment of Dysfunctional Breathing" was published in 2021. Journal: Front Physiol.

Moreover, many gaps remain in our knowledge that warrant further research. Despite the fact that erratic breathing patterns can be identified on CPET as discussed, CPET alone may not be able to sub-classify DB patients into the different sub-types. Further in-depth analysis of CPET data from patients with DB may help to elucidate patterns that define the different sub-types and thus improve our ability to classify DB. It may be that a combination approach using the patient’s history, assessment by a physiotherapist and CPET is required to classify DB.

In addition, CPET cannot currently directly quantify the degree of irregularity of the erratic breathing pattern. One small study has used calculation of approximate entropy to quantify ventilatory irregularity and was able to differentiate controls from patients with DB (Bansal et al., 2018). Though this technique requires further validation, it may prove useful not only for diagnostic purposes, but also as a way to quantify the severity of DB.

## Future Directions

Looking to the future, the implementation of CPET into standard clinical practice would greatly improve the diagnosis and management of DB. In the flowchart below, we provide an example as to where CPET can be incorporated into clinical practice to support the diagnosis of DB and subsequent therapeutic intervention (Figure 4). For dyspneic symptoms which remain despite obvious disease pathology being ruled out or optimized for, there should be a high suspicion of DB. CPET can then provide a useful method to investigate and confirm the presence of any abnormal breathing patterns, thus confirming the presence of DB.

**FIGURE 4:** Flowchart to illustrate a proposed clinical pathway for DB identification and therapy, based on current practice at Cambridge University Hospitals NHS trust. Suggested cut-off values are based on studies cited in this paper (Kinnula and Sovijarvi, 1993; Brat et al., 2019). FEV1, forced expiratory volume in 1 s; VeqCO2, ventilatory equivalent for CO2; P_*ET*_CO2, end-tidal CO2; *V*_*t*_, tidal volume; *B*_*f*_, breathing frequency.

The next steps may well be to improve CPET as a tool by targeting the limitations explained above. CPET, whilst being an attractive diagnostic method, currently cannot quantify the severity of DB, nor classify it into sub-types. Further study into potential ways to quantify and classify the DB using the CPET data should enhance the usefulness of the technique.

The article "Cardiopulmonary Exercise Testing in the Assessment of Dysfunctional Breathing" was published in 2021. Journal: Front Physiol.

Additionally, since it remains difficult to provide specific diagnostic cut-off values for DB, there may be a role for artificial intelligence to aid CPET interpretation in the future. Pattern recognition performed by an artificial intelligence system could identify erratic breathing, characteristic of DB, thereby simplifying the process of making a diagnosis. This may be an interesting avenue to consider as we look to refine CPET as a tool for the identification of DB.

Dysfunctional breathing is a condition driving significant symptom burden, which is difficult to characterize and yet has treatment options (Thomas et al., 2003). We have highlighted that the prevalence of DB is disproportionately high in patients with chronic disease such as asthma or COPD (Thomas et al., 2005) and that traditional diagnostic questionnaires may struggle to diagnose these cases of DB (Stanton et al., 2008). We encourage clinicians to consider the possibility of DB in those living with such conditions to avoid unnecessary and potentially harmful escalation of treatment.

Cardiopulmonary exercise testing represents the optimal modality of diagnosis of DB. In particular its ability to identify individuals’ functional capacity, as well as presence of concurrent disease, strengthens its clinical utility.

## Author Contributions

MI was primary author and was responsible for planning and putting together the first draft of the manuscript. MI, SM-B, LD-C, and CP contributed sections of the manuscript. JF, KS, MJ, and MI contributed figures. MJ contributed the table. All authors were involved in editing and finalizing the manuscript. JF oversaw and co-ordinated the process.

## Conflict of Interest

The authors declare that the research was conducted in the absence of any commercial or financial relationships that could be construed as a potential conflict of interest.
